The article "Research Progress on the Role of Inflammatory Mechanisms in the Development of Postoperative Cognitive Dysfunction" was published in 2021. Journal: Biomed Res Int.

# Research Progress on the Role of Inflammatory Mechanisms in the Development of Postoperative Cognitive Dysfunction

**DOI:** 10.1155/2021/3883204

**Published:** 2021-11-26

**Authors:** Xiao-xiang Tan, Li-Li Qiu, Jie Sun

**Affiliations:** Department of Anesthesiology, Zhongda Hospital, School of Medicine, Southeast University, Nanjing 210009, China

## Abstract

Postoperative cognitive dysfunction (POCD), as one of the common postoperative complications, mainly occurs after surgery and anesthesia, especially in the elderly. It refers to cognitive function changes such as decreased learning and memory ability and inability to concentrate. In severe cases, there could be personality changes and a decline in social behavior. At present, a great deal of research had been carried out on POCD, but its specific mechanism remains unclear. The release of peripheral inflammation-related factors, the degradation and destruction of the blood-brain barrier, the occurrence of central inflammation, and the neuronal apoptosis and synaptic loss could be promoted by neuroinflammation indicating that inflammatory mechanisms may play key roles in the occurrence of POCD.

## 1. Introduction

With the development of modern medicine, a growing number of elderly patients have the possibility to receive one or more life-extending surgical procedures [1]. However, postoperative cognitive dysfunction (POCD), as one of the common complications after surgery, had seriously threatened the quality of life especially for the elderly patients, extended the length of hospital stay, and increased the medical cost [2]. The international community is calling for systematic research on POCD, and there is an urgent need for reliable prediction and treatment methods [3, 4]. Until now, clinicians have not come to an agreement about POCD [5]. Postoperative cognitive dysfunction had been broadly defined as a significant decrease in cognitive ability following surgery or anesthesia [6]. Deficiency in neurological function included decreased executive ability, attention, verbal memory, intended motion, and visuospatial attraction [7]. Due to conflicting results and controversial evidence in different studies, the underlying pathogenesis of POCD remained unclear [8]. Many researchers had successfully established POCD models by intraperitoneal injection of lipopolysaccharide (LPS) to mice to induce neuroinflammation, and more attention had been paid to the mechanism of neuroinflammation caused by surgery or anesthesia in POCD animals [6, 9]. Neuroinflammation may be a common precursor of cognitive decline and was involved in the development of perioperative neurodegenerative diseases. Therefore, limiting acute neuroinflammation may ameliorate cognitive function, thus greatly improving patients' outcome [10]. This review will discuss the research progress of POCD from the perspective of inflammatory mechanisms.

## 2. POCD and Inflammation-Related Factors

Surgical trauma or anesthesia could increase the level of inflammatory cytokines in patients after surgery. Current studies on inflammation-related factors had focused on S100B protein, interleukin-6 (IL-6), interleukin-1*β* (IL-1*β*), interleukin-17 (IL-17), tumor necrosis factor-*α* (TNF-*α*), the complement system, inducible nitric oxide synthase (iNOS), cyclooxygenase-2 (COX-2), prostaglandin E (PGE), and other factors. And were the inflammatory cytokines from the surgical site or the local environment of the brain? The current view was basically the same. As described below, surgery resulted in an increase in inflammatory factors at the surgical site. Anesthesia could cause inflammation throughout the body as well as in the brain. The unique inflammatory cells of the brain, such as microglia, were activated in response to proinflammatory factors and promoted the progression of neuroinflammation. Each of these inflammatory factors will be described in the following paragraphs.

### 2.1. S100B Protein

As a member of the S100 family, the S100B protein belonged to calcium binding protein with low molecular weight of about 9-13 kDa [11]. It was a neurotrophic factor and neuronal survival protein during the development of the central nervous system [12] and could be released from damaged astrocytes in response to inflammation, ischemia reperfusion, and oxidative stress in the body [13]. Associated with many diseases, Alzheimer's disease [14], autoimmune diseases such as multiple sclerosis [15], psychiatric diseases such as schizophrenia [16], cerebrovascular diseases [17], and others, the S100B protein helped to enhance the interaction between neurons and glial cells [18] and indicated the severity of brain damage [19]. At the physiological level, the S100B protein stimulated neurite elongation, protected neuronal survival, and played a role in neuronal maturation and glial cell proliferation in vitro [20]. But some others showed a high level of neurotoxicity [21]. High concentration of the S100B protein stimulated the expression of proinflammatory cytokines, induced cell apoptosis, exerted its neurotoxic effect, and promoted the development of neurodegenerative diseases and neuroinflammation [22]. In some clinical studies, an association between S100B and POCD had been found. The S100B protein level was significantly elevated in POCD patients after total hip arthroplasty [23]. And in POCD patients after transurethral resection of the prostate under general anesthesia, its expression was significantly higher than those in patients without POCD [24]. Through investigating the relationship between POCD and the S100B protein level after robot-assisted laparoscopic radical prostatectomy (RALRP), it was concluded that S100B increased after RALRP, and this increase was related to the development of POCD [25]. At present, there is no consensus on whether the elevated expression level was an accompanying symptom, a cause, or a consequence. However, these researches may suggest that the degree of S100B protein concentration increase may be used as a biomarker for POCD and predict the occurrence of POCD after surgery and anesthesia.

### 2.2. Interleukin-6

IL-6 as an important signaling molecule in the immune system was an important regulator in synapse formation [26]. Under normal conditions, the IL-6 level in the central nervous system was usually low, possibly due to the low expression level of constituent in CNS cells. In some pathological ones, neurogliocyte [27] or neuronal stimulation significantly increased IL-6 levels in the CNS [28]. Locally, high concentrations of IL-6 could inhibit the synaptic function [29]. In adult transgenic rats overexpressing IL-6 in astrocytes, the hippocampal neuron in the dentate gyrus was reduced by 63% [29]. Neutralizing antibodies to IL-6 significantly improved long-term enhancement (LTP) and spatial memory in rats [30]. Besides, through rigorous regression analysis, the elevated plasma IL-6 level tended to be a risk factor leading to cognitive impairment [31]. This achievement further demonstrated that the role of IL-6 as a regulator was critical to cognitive function. More is needed to understand the conditions that the induction of IL-6 in the CNS and the therapeutic strategies that could ameliorate or promote the effects of IL-6.

### 2.3. Interleukin-1*β*

IL-1*β* was a potent proinflammatory cytokine produced by innate immune cells. The function of learning and memory in the brain depended on the proper functioning of the hippocampus, where IL-1*β* receptors were abundant [5, 32]. However, high levels of IL-1*β* were associated with decreased cognitive function [33]. Besides, some studies have shown that increased levels of IL-1*β* in the inflammatory response induced by LPS in mice aggravated the cognitive impairment following anesthesia and surgery [34]. Overexpression of IL-1*β* also induced the alteration of microglial gene expression profile and microglial expansion and promoted neuroinflammation [35, 36]. Although there were few studies on the direct relationship between IL-1*β* and POCD, the important role of IL-1*β* in neuroinflammatory response suggested that it may be a reminder of its importance in POCD.

### 2.4. Interleukin-17

IL-17, an early promoter of T cell-induced inflammatory response, not only was an important member of the body against infection but also was closely related to the regulation of autoimmunity [37]. It could exacerbate inflammation by inducing the secretion of proinflammatory cytokines, such as IL-1*β*, IL-6, and TNF-*α* [38]. And in the development of multiple sclerosis and cerebral hemorrhage, some research had suggested that IL-17 was involved in the inflammatory response [39, 40]. It had also been found to promote the breakdown of the blood-brain barrier and the transfer of inflammatory mediators from the periphery to the center [41, 42]. Another piece of evidence had shown that blocking IL-17 alleviated cognitive impairment due to inflammation caused by surgical trauma [43]. In a clinical investigation, the serum IL-17 concentration of patients with Alzheimer's disease (*P* = 0.0023) was significantly higher than those of the control group [44]. In animal studies, IL-17 was involved in LPS-induced neuroinflammation and cognitive impairment in elderly rats through microglial activation [45]. Anti-IL-17 treatment improved oxidative stress and neuroinflammation and ultimately alleviated cognitive impairment in sevoflurane anesthetized elderly rats [46]. These above achievements hinted that anti-IL-17 may represent a novel therapeutic strategy for neuroinflammation and POCD.

### 2.5. Tumor Necrosis Factor-*α*

TNF-*α* was a protein involved in the signaling of immune response cells, which could promote the inflammation [47, 48]. In the inflammatory response, TNF-*α* increased the production of other proinflammatory cytokines, such as IL-1, IL-6, and IL-8 [49]. TNF-*α* was also involved in many physiological processes in the central nervous system [50]. The presence of a large number of cytokine receptors in the hippocampus during neuroinflammation made it susceptible to high concentrations of proinflammatory cytokines, such as TNF-*α* [51, 52]. Once these cytokine receptors were activated at high levels, the metabolic Glu2 receptors were downregulated to enhance the AMPA/NMDA signaling which could disrupt the LTP process [53]. In addition, TNF-*α* restrained inhibitory neurotransmission by downregulating GABA receptors, disrupted the delicate balance between excitatory and inhibitory neurotransmission, and ultimately promoted the glutamate toxicity [54]. It had contributed to the advancement of cognitive dysfunction. In these completed studies, isoflurane anesthesia increased the incidence of POCD in diabetic rats through the TNF-*α*-dependent mechanism [55]. After undergoing elective head and neck cancer surgery under general anesthesia, the postoperative TNF-*α* level was obviously increased in the POCD group [56]. The group with the highest TNF-*α* level had a significantly higher incidence of POCD than the control group undergoing unilateral hip replacement [57]. Although there were so many studies proving the corelationship between TNF-*α* and POCD, the mechanism by which TNF regulated the progression of POCD was still unclear.

### 2.6. The Complement System

The complement system consisted of more than 30 proteins that had long been known to be involved in immune defense against pathogens and the removal of damaged cells. In the central nervous system, complement proteins were widely expressed in neurons and glial cells, and studies had shown that microglial cell-mediated synaptic phagocytosis depended on the CR3/C3 (complement receptor 3/complement 3) [58]. More importantly, some research found that CR3 was a phagocytic receptor on the surface of microglia and was specifically expressed in the brain by microglia [59]. As a CR3-recognized ligand, complement C3 was located in synapse-rich regions of the brain and guided microglia to recognize the phagocytosis [60]. It had been shown that the level of complement protein in the hippocampus was high before the deposition of *β*-amyloid (A*β*) and cognitive deficit in Alzheimer's disease model mice [61, 62]. Complement proteins had been localized to the synaptic element before the synapse was lost [61]. Furthermore, when the C3 or CR3 gene was knocked out, the microglia phagocytosis of synaptic structure was significantly reduced, the synaptic structure was protected, and the cognitive function of mice was also significantly improved [62, 63]. Therefore, the regulation of complement signals may have the potential to be a new treatment strategy for POCD.

### 2.7. Inducible Nitric Oxide Synthase

Nitric oxide synthase (NOS) was an isoenzyme which was classified into neuronal nitric oxide synthase (nNOS), endothelial nitric oxide synthase (eNOS), and inducible nitric oxide synthase (iNOS) [64]. As a participant in inflammation, iNOS did not appear under normal condition and could be expressed by the stimulation of endotoxin LPS and a variety of cytokines, such as TNF-*α* and IL-1 [65]. It could promote synaptic plasticity and brain deficits, such as cognitive deficits [66]. Furthermore, as a product of NOS, nitric oxide (NO) played a crucial role in supporting normal physiological functions [67], but pathological conditions such as inflammation could stimulate high levels of the NO production which may trigger neurodegeneration [68, 69]. L-Nitroarginine methyl ester was a NOS inhibitor that could inhibit NO biosynthesis and alleviate brain dysfunction [70]. By reversing the NO signaling pathway, cognitive deficits and inflammatory responses in mice induced by carotid artery exposure surgery were alleviated [71]. Therefore, NO was considered to be a predictive risk factor for Alzheimer's disease (AD) and early POCD [72].

### 2.8. Cyclooxygenase-2 and Prostaglandin E

Cyclooxygenases were a group of heme-containing isoenzymes (COX-1 and COX-2) that catalyzed the conversion of arachidonic acid to the primarily bioactive prostaglandin (PG) [73]. COX-2 was constitutively expressed in the postsynaptic dendrites and excitatory terminus of cortical and spinal neurons in the brain [74]. And most of the focus of COX-2 induction had been on neurodegenerative and psychiatric disorders associated with neuroinflammation [74] and promoted the progression of POCD to a certain extent [75]. Then, it could produce PGE2 in response to synaptic activation. PGE2 may undergo retrograde transport across the synapse, stimulate glutamate release from presynaptic neurons by activating the presynaptic Ep 2 receptor from the postsynaptic [76]. The increase of glutamate release reduced the number of small albumin-positive GABA cells [77]. PGE2 had the ability to become a key messenger of COX-2-mediated synaptic transmission and plasticity regulation in the hippocampus [78]. On the side, PGE2 stimulated microglia, astrocytes, and neurons to produce amyloid (A*β*) in vitro and in vivo [79]. As we know, it was detrimental to brain function. These previous studies had shown that COX-2 was involved in synaptic transmission and plasticity while Prostaglandin E2 (PGE2), a key molecule in COX-2-mediated synaptic modification, played an indispensable role. Although these were not directly related to POCD, they did bring us some enlightenment.

## 3. POCD and the Blood-Brain Barrier

In general, the blood-brain barrier (BBB) was mainly composed of the glial membrane, which consisted of the terminal foot of astrocytes, capillary basement membrane, and capillary endothelial cells [80]. Three layers of structures were closely connected [81]. This compact structure allowed only water, gases, and small fat-soluble molecules to passively spread across the BBB [82]. However, proinflammatory cytokines such as IL-1 and TNF-*α* could upregulate COX-2 in neurovascular endothelial cells, thereby promoting local prostaglandin synthesis and impairing BBB permeability [10, 83]. TNF-*α* also upregulated the transcription of matrix metalloproteinase (MMP), especially MMP-9 which degraded extracellular matrix proteins and further decomposed the BBB [81]. MMP-9 deletion mice which were exposed to surgical trauma showed better cognitive performance in terms of fear conditions compared to the wild-type mice [84]. In the case of central nervous system (CNS) inflammation and subsequent BBB breakdown, bone-marrow-derived monocytes (BMDM) were recruited to CNS through an interaction between chemokine monocyte chemical attractor protein 1 (MCP-1) and BMDM cell surface [85]. Once BMDM was present in the CNS, it continued to secrete proinflammatory cytokines by upregulating NF-*κ*B transcription [86] and activated microglia cells to further amplify the neuroinflammation. In mouse models, the occurrence of POCD was reduced by preoperative depletion of BMDM [87]. It suggested that BMDM migration may play a key role in POCD. Therefore, it was believed that once the BBB was destroyed, cytokines took the opportunity to enter the CNS freely, led the transport of BMDMs to nervous tissues, and initiated the state of dysregulation of immune function. The immune system in the central nerve system was linked to the periphery through the blood-brain barrier, which aggravated the neuroinflammatory response, brain tissue damage, and development of POCD.

## 4. POCD and the Gut-Brain Axis

Intestinal microflora mainly existed in the digestive tract and was an important part of the human microflora. A great many of animal and human research evidence suggested that brain function and microenvironment were largely influenced by gut microbes through hormones, immune molecules, and the specific metabolites they produced [88]. The connection between gut microbes and the brain was known as the gut-brain axis [89]. The gut-brain axis was a two-way communication system between the central nervous system (the brain) and the gut [90]. An array of bacteria, viruses, and other microbes made up the gut microbiome. Dysregulation of intestinal flora may contribute to the progression of neurodegenerative diseases and promote the release of inflammatory markers such as TNF-*α* and IL-6 [91, 92]. Some studies found that AD patients were often accompanied by intestinal flora disorders, increased BBB permeability, and promoted large amounts of bacterial amyloid protein and lipopolysaccharide into the circulatory system and CNS, ultimately leading to cognitive impairment [93]. Mice on a high-fat diet also showed increased systemic and CNS inflammation, which in turn resulted in reduced cognitive function by affecting the gut-microbiota–gut-brain axis system [94]. Bifidobacterium as an “immune organism” could beneficially regulate neuroinflammatory response and behavior in many models of neuroinflammation-related diseases [95, 96]. Lactobacillus, another widely studied microbial strain, effectively protected against memory deficits and neuroinflammation in aging mouse models with Alzheimer's disease [97, 98]. Therefore, intestinal flora had been increasingly studied as a key regulator of neuroinflammation. Galactose oligosaccharide (B-GOS) blends were well-studied specific nondigestible galactose oligosaccharides. In particular, it selectively promoted the proliferation of bifidobacterium [99]. Other experiments had also revealed that B-GOS inhibited the overactivation of microglia and decreased the proportion of microglia of the M1 phenotype induced by surgery. In addition, B-GOS feeding exerted a sufficient prebiotic effect in promoting the proliferation of potential anti-inflammatory microorganisms which may contribute to the regulation of surgically induced neuroinflammatory responses via the microbiome-brain axis [100]. Fecal filtrate from healthy people was injected into the intestinal tract of patients with neurological diseases to increase the number of beneficial bacteria and reduce the number of harmful bacteria to maintain the homeostasis of intestinal flora inpatients [101]. Dysregulation of intestinal flora could contribute to the progression of neurodegenerative diseases. Thus, regulation of the intestinal microbiota may be a potential treatment for various neurological diseases [102]. Although these measures had not yet been rolled out effectively, they offered an opportunity to intervene in the disease progression.

## 5. POCD and Microglia

Microglia, as the innate immune effector cells in the CNS, had the characteristics of multiple synapses and plasticity and played an extremely important role in the physiological process of the CNS [103, 104]. Normally, the CX3CR1 protein in the brain bound to the microglia CX3CR1 receptor, inactivating microglia [105]. When inflammation, infection, trauma, or other neurological diseases occurred in the brain, microglia cells, the first responders of pathogens in the CNS, were rapidly activated and gained the phagocytic function. They could affect the synaptic connections between neurons and promote neuroinflammation [106]. Activated mast cells (MCs) may also induce microglial activation and neuronal damage leading to inflammation of the CNS [107]. Inactive microglia could be activated and differentiated into one of two phenotypes, M1 or M2 [108]. The M1 phenotype was highly phagocytic and proinflammatory, while the M2 phenotype was anti-inflammatory and involved in tissue repair and remodeling [109, 110]. Proinflammatory mediators (TNF-*α* or LPS) promoted the differentiation of microglia into the M1 type, while anti-inflammatory cytokines (IL-4) promoted the expression of the M2 phenotype [111]. Microglia activated differentiation to the M1 type, leading to continuous expression of proinflammatory cytokines which amplified neuroinflammation and accelerated the development of POCD [112, 113]. In various experimental animal models, activated microglia released HMGB1, TNF-*α*, and IL-1*β* [114]. These chemokines promoted the further flow of BMDM into CNS, while the transported BMDM continued to activate microglia to the M1 phenotype. Besides, perioperative microglia depletion [112] and promotion of M2 phenotype expression in mice research through the administration of erythropoietin [115] improved both memory and cognitive dysfunction. This further confirmed that microglia may play an important role in the mechanism of POCD. The characteristics of microglia in the elderly human brain were malnutrition with increased expression of inflammatory markers, decreased expression of neuroprotective factors, decreased ability of migration and clearance, decreased ability to regulate injury and recovery, and changed from the anti-inflammatory state to the proinflammatory state [116]. These changes underlay an increased susceptibility to neurodegenerative changes in the elderly. Although previous studies found that microglia activation played a key role in the pathogenesis of POCD, the core mechanism of how microglia affected neuronal function and led to cognitive decline was still unclear.

## 6. POCD and Neurons and Synapses

The density of synapses decreased with age in humans and other mammals, but not all brain regions were equally sensitive to aging [117]. The changes were more pronounced in the prefrontal cortex and hippocampus than in other brain regions [118, 119]. Lack of neuronal activity or cell death caused synapses to malfunction and led to neurodegenerative diseases [120]. Neurons must undergo drastic structural changes to become presynaptic or postsynaptic. Synapses were structures that strengthened the connections between neurons and a cross-cell unit composed of presynaptic membrane, synaptic cleft, and postsynaptic membrane. Because of this particular composition, they transmitted information between neurons effectively [121]. Newly formed synapses were not static, as they underwent constant change in order to meet their behavioral needs in a constantly changing environment [122]. These changes could be in the formation of new synapses or in the enhancement of synaptic efficacy known as synaptic plasticity [123]. Inflammatory cytokines produced by surgical or anesthetic factors crossed the BBB and entered to the CNS to cause the central inflammatory cell activation. These inflammatory cells would continue to release a series of pathological proteins such as inflammatory cytokines, injurious proteins, and neurotoxins, which could interact with neurons and synapses, resulting in neuronal death, synaptic loss, and the inability of cell signaling, eventually leading to the occurrence of POCD [124]. Possible mechanisms were as follows: (1) Phosphorylated Tau protein and synaptic terminal A*β* plaques [125] aggregated in neurons, destroyed the structure of surrounding neurons and synapses, and injured the signaling function. (2) TNF-*α* [126] released by glial cells and IL-16 [127] from lymphocytes could lead to intoxication by inhibiting the metabolism and over accumulation of glutamate. GABA receptors were downregulated to inhibit inhibitory neurotransmission, such as parvalbumin (PV) neurons, an important class of inhibitory interneurons in GABA-capable neurons, which could disrupt the balance between excitatory and inhibitory neurotransmission and reduce neuronal excitability and synaptic activity [54]. (3) Activation of inflammasome NLRP3 only in microglia depended on JNK1-mediated dephosphorylation of S194 [128]. Mitochondria-derived reactive oxygen species (MTROs) produced after surgery or anesthesia not only acted as upstream NLRP3 activators but also participated in the assembly of downstream inflammasomes [129]. Mitochondria, as the main site of reactive oxygen species (ROS) production, were most vulnerable to ROS attacks. After oxidative damage, the mitochondrial respiratory chain was destroyed and a vicious cycle was formed which eventually led to nerve apoptosis [130]. Generally speaking, the damage of neurons and the decline of synaptic plasticity were the most fundamental factors leading to POCD. This should be universally acknowledged. Therefore, how to intervene to reduce the loss of neuronal and synaptic function will be the focus of future research.

## 7. Possible Prevention and Therapeutic Ways

The neuroinflammatory hypothesis offered many different directions for candidate treatment of POCD. By blocking various links of the inflammatory response, the blocking of neuroinflammatory response had produced positive effects in clinical or animal experiments.

Dexamethasone, as a synthetic glucocorticoid, had a powerful anti-inflammatory effect. Meanwhile, anti-inflammatory effects in brain cells had been demonstrated in several studies [131, 132]. Postoperative inflammatory response syndrome could be suppressed by using large doses of dexamethasone during the cardiac surgery [133], and patients receiving dexamethasone underwent shorter hospital stays and a lower risk of postoperative delirium and infection [134]. In noncardiac and nonneurological procedures, dexamethasone reduced the incidence of POCD in elderly surgical patients when BIS was associated at 46–55 [135]. In sevoflurane-induced cognitive impairment in adult rats, the addition of dexamethasone improved short-term and long-term cognitive impairment in adult rats and reduced the expression of the inflammatory cytokine IL-6 [136].

Cox-2 was constitutionally expressed in the brain and involved in the development of neuroinflammation by catalyzing the conversion of arachidonic acid into the proinflammatory prostaglandins [83]. It could increase the blood-brain barrier permeability to promote the entry of inflammatory factors into the brain [10]. Therefore, COX-2 inhibitors were considered as important interventions for neuroinflammation and potential targets for treatment of POCD. Celecoxib, a highly selective COX-2 inhibitor, significantly reduced the incidence of POCD and plasma levels of IL-1*β*, IL-6, TNF-*α*, COX-2, and S100B on day 7 after total knee replacement in elderly patients, although there existed no difference in the incidence of POCD between the two groups after 3 months [137]. Parecoxib inhibited the overexpression of COX-2 and decreased the levels of IL-1*β*, IL-6, TNF-*α*, and PGE2 in the brain of rats. The cognitive function of POCD rats was improved [138]. Intraperitoneal injection of the COX-2 inhibitor meloxicam 24 h after splenectomy prevented surgically induced cognitive dysfunction and inhibited glial cell activation in mice [139]. Cox-2 inhibitors had not been particularly fully studied for cognitive improvement, while many studies proved a possible solution.

Minocycline was a broad-spectrum antibacterial tetracycline antibiotic that could easily cross the blood-brain barrier (BBB) to exert anti-inflammatory effects [140]. It has been proven that minocycline played a neuroprotective role by inhibiting inflammatory responses and reducing neuronal apoptosis [141]. In isoflurane or surgery-induced cognitive impairment models, it was found that minocycline could downregulate microglia marker IBA-1 protein expression [142] and upregulate anti-inflammatory cytokine IL-4 and IL-10 protein levels [143]. The pretreatment of minocycline enhanced spatial orientation memory in elderly mice by inhibiting microglial activation and reducing the release of proinflammatory cytokines in the hippocampus [144]. Other study also showed that minocycline successfully reduced the cognitive impairment associated with LPS-induced neuroinflammation and decreased the production of neuroinflammatory markers in the hippocampus and cortex [145]. Being a key link in the induction of neuroinflammation, microglia had been demonstrated in Alzheimer's disease [146]. Strategies targeting microglia provided an interesting area for further research into the prevention and even treatment of POCD. In a mouse model, perioperative microglial depletion [112] and promotion of the M2 phenotypes by injection of erythropoietin [115] all improved the memory dysfunction which were verified in passive avoidance and new object recognition tests. In a recent rat study, peripheral surgery induced CNS mast cell degranulation and subsequent microglial activation [147]. The use of sodium glycyrrhea reduced the degranulation of mast cells and inhibited the activation of microglia in rats, thus improving the memory ability [148].

As a key regulator of neuroinflammation, gut microbiota could regulate host immunity and cognition [149]. Therefore, the regulation of gut microbiota may be a potential treatment for various of neurological diseases [102]. Prebiotics could be selectively utilized by host microbes to stimulate the gastrointestinal microbiota and confer health benefits [150]. A growing body of evidence indicated that the contained prebiotics diet was beneficial for the host immune and gut-brain shaft. It helped to reduce the nerve inflammation [151]. Surgical trauma and anesthesia altered the composition of the gut microbiome. Neuroinflammatory response and spatial learning and memory disorders could be alleviated by preconditioning with SCFA (metabolites of intestinal microorganisms [152]).

Anesthesia and surgery created inflammation of the body. Appropriate inflammatory response could inhibit the harmful factors and facilitate the rapid recovery of the organism. Excessive inflammatory response and the inability of inflammatory factors to distinguish between enemy and self led to the disorder of neuronal function and promoted the development of POCD. The intervention of various of stages of inflammation occurrence and development had achieved encouraging positive results. These studies had laid a firm foundation for a more comprehensive intervention and even treatment.

## 8. Conclusions

The morbidity of POCD was particularly prominent in the elderly, and the increase of postoperative mortality made it urgent to understand the pathogenesis. Involvement of inflammation-related factors and microglia activation had been shown to play a role in cognitive decline, while some inflammatory factor receptor antagonists and drugs may ameliorate the cognitive decline after surgery. The interaction between the peripheral immune system and the CNS was also involved. The role of inflammatory mechanisms in the development of POCD was briefly illustrated in Figure 1. But the current results were not enough to shed light on how activated glial cells modulate neuronal transmission and how they changed the synapses that could affect neuron function. Clinical and primary medical professionals are working hard to explore the pathogenesis of POCD, develop effective drugs, or improve surgical techniques to treat or prevent POCD. Although it may need more time to find new predictors and therapeutic targets, continuous researches and explorations are expected to pave the way for standardized treatment for POCD and bring good news to POCD patients.

## Figures and Tables

**Figure 1:** Flowchart of inflammatory mechanisms. The picture shows that after anesthesia or surgery, the activation of multiple inflammatory and proinflammatory cytokines, as well as the reduction of BBB function, promoted the transfer of inflammation-related factors from the periphery to the center. With the neuroinflammation progressing, the function of neurons in the brain continued to decline over time. And the presence of the gut-brain axis also played a key role in the transport of these cytokines. Consequently, the inflammatory mechanism of POCD was a combination of multiple factors. Abbreviation: IL-1*β*: interleukin-1*β*; IL-6: interleukin-6; IL-17: interleukin-17; TNF-*α*: tumor necrosis factor-*α*; iNOS: inducible nitric oxide synthase; COX-2: cyclooxygenase-2; PGE: prostaglandin E; MMP: matrix metalloproteinase.
